# Music Art Teaching Quality Evaluation System Based on Convolutional Neural Network

This article has been retracted.

**DOI:** 10.1155/2022/8479940

**Published:** 2022-06-02

**Authors:** Fumei Xu, Yu Xia

**Affiliations:** ^1^School of Music, Jiangxi Normal University, Nanchang Jiangxi 330027, China; ^2^School of Aviation Services and Music, Nanchang Hangkong University, Nanchang Jiangxi 330063, China

## Abstract

With the rapid growth of music and art education in colleges and universities today, the development of associated teaching quality assessment (TQE) is still in its infancy. In truth, most modern music and art education has yet to build a rigorous and appropriate evaluation system based on actual classroom teaching quality. Simply adopting classroom TQE indicators and approaches from other disciplines would unavoidably lead to formalization of music TQE findings in some schools and institutions. It has no bearing on evaluation, feedback, or advancement. Therefore, this paper uses the superior performance of neural network to solve nonlinear problems and constructs a music art TQE method based on convolutional neural network (CNN). The completed work is as follows: (1) The basic situation of domestic and foreign research on music art TQE is introduced. Several commonly used TQE methods at home and abroad are analyzed, and the CNN evaluation method is comprehensively introduced. (2) The principle and network structure of CNN are expounded, and a TQE system conforming to music art is constructed. (3) The final experimental results reveal that the CNN model has higher accuracy and better performance than the BP neural network when using the trained CNN, TQE model to conduct tests.

## 1. Introduction

My country's general higher music education started early, but in the 1960s and 1970s, due to the influence of many factors such as history, the development was relatively slow. The formulation and promulgation provided stronger theoretical support for the development of music education and pointed out the direction for the revitalization and development of music education [1, 2]. It emphasizes the status and role of art education in school education. According to the strategy, schools should emphasize art instruction as a key component of a broader effort to promote aesthetic sensibility among students. A powerful means of intellectual and physical health development, art education, as an important part of school education, has an irreplaceable role in other disciplines [3]. China's college music education is booming today, but some aspects of its construction are still immature. For example, music classroom teaching objectives, teaching content selection, teaching methods, and teaching effect evaluation have different degrees of defects in classroom teaching performance and research. How to optimize the evaluation theory and practice of music classroom teaching is the top priority of current college music education. In fact, most of the current music teaching has not really established a scientific and reasonable evaluation system based on the actual teaching quality in the classroom [4]: for example, what kind of teaching configuration is required for music teaching in colleges and universities and what kind of TQE system is required, rather than just blindly copying the TQE indicators and models of other disciplines or any subject in the school, which will inevitably lead to some college music teaching. The results of evaluation are only a form and do not play a real role in evaluation, feedback, and promotion. Therefore, the research on the TQE system of music classroom teaching still needs to carry out research methods that are in-depth and systematic, combining theory and practice, so as to recognize the key elements of college music TQE in essence [5]. Music education is a music education subject for ordinary college students who are not majoring in music, including classroom teaching, music art practice, campus music and cultural activities, and other educational forms. Because of its strong systematic teaching content, wide knowledge coverage, strong knowledge compatibility with related art and cultural fields, regular learning cycle, gradual knowledge difficulty, and ability to be carried out for many college students at different levels, music classroom teaching has become an important part of music classroom teaching. This is the most common method of music teaching in schools for ordinary college students [6]. The method of summative evaluation that formerly concentrated on results and overlooked the process has evolved to some extent in the evaluation of music classroom teaching. However, in view of the current situation of higher education, students can enter colleges basically through exam-oriented education. Such students have long been accustomed to the performance-based educational evaluation model. One of its consequences is that it is difficult to apply formative evaluation methods to classroom teaching evaluation. The TQE of music classroom should not only conform to the laws and characteristics of music art education and teaching but also combine the inherent characteristics of popular education and teaching. It should not only reflect the essential factors of classroom teaching work but also take into account the purpose and characteristics of popularization of teaching [7]. The activity of music education and instruction should be guided and promoted by evaluation indicators, and this may be considered a balance. Continuous development in the quality of education and instruction can only occur in this manner. TQE for music and art based on CNN is proposed in this study, following this backdrop, and uses the advantages of neural networks to solve nonlinear problems to find a more suitable teacher's TQE method and model for music and art education. The methodology eliminates the impact of human variables on the assessment outcomes, and the rational teaching evaluation offers a useful reference for the investigation of other areas of teaching evaluation.

The paper's section-by-section study paragraph is as follows: The related work is presented in Section 2.  Section 3 analyzes the methods of the proposed work.  Section 4 discusses the experiments and results. Finally, in Section 5, the research work is concluded.

## 2. Related Work

In the teaching thinking and exploration of music teaching method courses in colleges and universities, Reference [8] takes microteaching method and example teaching method as the breakthrough point and proposes how to train the basic skills of college students. On the one hand, it proposes to strengthen the basic knowledge of music. To study, we must also strengthen the training of basic teaching skills of college students. Only in this way can we solve the current situation of low teaching ability of graduates. In addition, the weak basic knowledge of music education theory and the lack of basic skills of music teaching are also the main problems that should be solved in music teaching in colleges and universities. Reference [9] focuses on research on theoretical music teaching. Calling on music education in normal schools not only introduces music pedagogy but also pointed out that there is a lack of teaching books for teachers and professional music teaching materials. Music teaching methods are generally the teaching experience of teachers themselves, lacking the theoretical guidance and scientific nature of pedagogy. It is suggested to incorporate teaching methods into the music pedagogy system in colleges and universities. Reference [10] explores how to optimize the classroom structure and how to improve the teaching effect of music class from the macro- and microlevels and analyzes its structure. Reference [11] advocates an eclectic and comprehensive teaching method in terms of teaching methods. It is thought that instructional materials should be methodical and scientific, adaptable and practical, ideological and national, and practical and fundamental. Since 2000, some key domestic universities and teachers have started to construct TQE systems, and the long-term application of the results has promoted other universities [12]. A normal university started to develop a TQE system in 2002. A public database platform was established. The establishment of the online evaluation system promoted teachers' and students' information feedback system and multiple management information aggregation systems based on public data platforms [13]. Our country has obtained the campus network TQE system of the majority. With the informatization of education, according to the latest information of the National Education Informatization Construction Work Conference, the introduction of new IT technology will apply positive and effective evaluation technology to modern education through the system and create favorable conditions for the leap-forward development of the information of the evaluation system of college teachers [14].

The current TQE system adopts different evaluation methods and index systems according to the specific implementation of different teacher evaluation systems. By strengthening the school's information technology, it realizes the management of the teaching and research environment with a high degree of resource sharing. Through reasonable allocation, the digitization and information networking of teaching management and scientific research service evaluation on campus can be realized, the safety, reliability and scientificity of the system can be ensured, and the reasonable planning of services and feedback information mechanism can be used to realize resource complementarity and further improve the school management process and quality on the management system, assuring efficiency and effectiveness [15]. Examine renowned universities from throughout the world, such as those in California. Every year, three exceptional teacher awards are given out by Berkeley's world-class research institution to teachers who have made noteworthy achievements based on teaching assessment reports. The Berkeley teacher assessment system [16] consists of teachers' self-evaluation, mutual evaluation, and student evaluation. Foreign countries completely broke the traditional learning management system before the 1990s, and the evaluation system has used computers to improve the management level and strive to improve the best TQE system possible, which will surpass the business process to improve teaching and work efficiency [17]. As personal computers and local area networks became more common in the early 1990s, the TQE system began to use computers to change from mechanized business processes to scientific business processes, utilize the potential of modern information technology, and fully, more rationally, and effectively evaluate, which makes the school's teaching management more simplified. Subsequently, information technology has better penetrated into education and teacher evaluation, the rapid popularization of the Internet, and the wide application of the Internet, TQE has become the field of the Internet era [18, 19]. In the past two decades, in addition to the information resources provided by the Internet in classroom teaching, students and teachers have established a systematic interconnection system. Various services are implemented by students in computer networks. At the same time, using the Internet to surf the Internet also enhances the interaction between teachers and schools. Students, schools, and teachers establish strategic partnerships that provide new technological support in the information age, enhancing communication and interaction between them [20–22]. In today's Internet era, TQE also adopts a method that combines artificial intelligence technology to continuously develop and improve a better school evaluation mechanism. Neural network technology can upgrade the existing system structure to an advanced scientific evaluation system.

## 3. Method

In this chapter, we define the convolutional neural network structure, building a CNN prediction model and constructing a quality assessment system for music and art teaching in detail.

### 3.1. Convolutional Neural Network Structure

The layers of a basic CNN are often organized in a certain sequence. The data is transmitted from one layer to the next using a differentiable activation function at each node in the network. These layers include convolutional and activation layers as well as pooling and fully connected. It is possible to build a whole network by stacking these layers. Among them, the convolutional layer can affect the characteristics of the network, and the pooling layer affects the robustness of the network. The convolutional layer and the pooling layer together form a feature extraction layer for feature extraction.

#### 3.1.1. Convolutional Layers

To build a CNN, you need a convolutional layer at the very bottom. Local connections and weight sharing enable it to be much larger than a standard neural network since it is responsible for the majority of the network's processing. The number of weights and the number of trainable parameters are reduced, the problem of overfitting caused by too many parameters is avoided, the local perception area is effectively used, and the memory required for operation is reduced. Different input characteristics are retrieved by the convolution process, which is mostly executed in the convolution layer. The convolution operation is that the convolution kernel travels upstream of the input data with a certain step size, the weight of the convolution kernel is multiplied by the corresponding element of the traveled position, and the obtained results are added to obtain a new value as the output until the travel. Stop when all regions of the convolutional layer are finished. Its calculation formula is as follows:

(1) $$\begin{array}{c} y_{i}=f\left(\overset{n}{\underset{i=1}{\sum }}w_{i}x_{i}+p\right), \end{array}$$

where *y*_*i*_ represents the result after convolution calculation, *w*_*i*_ represents the weight of the convolution kernel, *x*_*i*_ represents the locally convolved area, and *p* represents the bias. The convolution kernel multiplies the input data, adds the multiplied results, and utilizes the added result as the output during a convolution process. The end result of the convolution kernel traversing the full input data will output a feature matrix to the following layer.

#### 3.1.2. Activation Layer

In the CNN structure, the activation function in the activation layer connects the convolutional, pooling, and fully connected layers in order. The activation function in the activation layer cannot be used to activate a neuron; rather, the function is used to maintain and transfer the active neuron characteristics to another space, with the goal of improving the features' linear separability. At present, the commonly used activation functions mainly include the following three functional forms: Sigmoid function, tanh function, and ReLU function. The specific formulas are as follows:

(2) $$\begin{array}{c} f\left(x\right)=\frac{1}{1+e^{-x}}, \end{array}$$

(3) $$\begin{array}{c} f\left(x\right)=\tanh\left(x\right)=\frac{e^{x}-e^{-x}}{e^{x}+e^{-x}}=2\mu \left(2x\right)-1, \end{array}$$

(4) $$\begin{array}{c} f\left(x\right)=\max\left(0,x\right)=\left\{\begin{array}{c} 0,\;x<0,\\ x,\;x\geq 0. \end{array}\right. \end{array}$$

Therefore, it is hoped that the activation function must have nonlinear characteristics and be continuously differentiable to meet the requirements of gradient descent, while satisfying the condition that the gradient is not saturated in the range. Since the calculation speed of the sigmoid function is slow and the derivative value is small, the maximum value is only 1/4. When the input value is high or small, the derivative approaches zero, resulting in network back-propagation. The quick decay of the gradient reduces or even eliminates the gradient communicated to the previous layer, making network training extremely challenging. Gradient dispersion is another name for this phenomena. Similarly, the tanh function also has the problem of gradient saturation. Therefore, these two activation functions are less used at present. For the ReLu function, when *x* > 0, the gradient is always 1, which avoids the problem of gradient dispersion and at the same time converges faster; when *x* < 0, the output is 0 and the training result is 0. The more neurons, the sparseness of the network becomes larger, the stronger the extracted features, the stronger the robustness of the network, and the faster the operation rate. Because of the above advantages, the ReLU function has now become the first choice for the CNN structure.

#### 3.1.3. Pooling Layer

It is common practice to include a pooling layer between convolutional layers in order to minimize both the number of parameters and data size, hence enhancing resilience of features and successfully avoiding overfitting. In the pooling layer, the main operation is the pooling operation or the downsampling operation, so the pooling layer is also called the downsampling layer. The most commonly used downsampling methods mainly include max pooling and mean pooling, and the specific formulas are as follows:

(5) $$\begin{array}{c} P_{m}=\underset{d+1\leq n\leq md}{\max}\left\{x_{n}\right\}, \end{array}$$

(6) $$\begin{array}{c} P_{a}=\frac{1}{w}\overset{md}{\underset{n}{\sum }}x_{n}, \end{array}$$

where *P*_*m*_ is the value after max pooling, *P*_*a*_ is the value after mean pooling, *d* is the width of the pooling filter, and *x*_*n*_ is the *n*th element in the pooling area.

During the pooling procedure, the filter is used to traverse the whole data set with a predetermined step size. When using a filter, it is best to utilize maximum and mean pooling, respectively, so that the pooled value of the area is equal to the sum of the area's values. As a result, the region's average is used as the pooled value. As of now, the vast majority of pooling in applications is maximum pooling, which provides location-independent characteristics.

#### 3.1.4. Fully Connected Layer

Each node in the fully connected layer is linked to all nodes in the previous layer, and the front-end features are combined to connect all of the features. The specific formula is as follows:

(7) $$\begin{array}{c} f=p_{j}+\overset{j}{\underset{m=1}{\sum }}w_{m}z_{m}, \end{array}$$

where *p*_*j*_ represents the bias matrix and *w*_*m*_ is the weight matrix, which describes the contribution of *z*_*m*_ to the output. The fully connected layer expands the output results obtained after pooling in turn into a one-dimensional feature vector and fully connects the feature vector with the output layer and finally outputs the result.

### 3.2. Building a CNN Prediction Model

Convolutional, pooling, and fully linked layers make up the bulk of the CNN. The number of convolutional layers, as well as the size, number, and stride of the convolution kernels in each convolutional layer, makes up the majority of the CNN structure. Other aspects, such as how many pooling layers there are and how they are sized, the activation function, the fully connected layer classifier, and other parameters are decided. In this section, for the planetary gear fault, the selected parameters are used to build the network structure, and the network model is trained at the same time, and finally, the construction of the CNN network prediction model is completed.

#### 3.2.1. Determination of Input Sample Data Format

In the field of TQE research, different from the two-dimensional input or time series data input generally used in CNNs, the data for TQE is a one-dimensional *N* × 1 data form. As a result, there are two types of input data: one-dimensional input, which involves directly entering the collected raw data, and two-dimensional input, which involves folding the one-dimensional data to maintain the overall quantity of data. In this case, the one-dimensional data is converted into a two-dimensional matrix input in the form of picture data, and the one-dimensional input form is selected in this paper.

#### 3.2.2. Build the Network Structure

First, build the model network structure. This section intends to build a 3-layer deep network structure with 2 convolution layers, 2 pooling layers, and a fully connected layer. The schematic diagram of the network structure is shown in Figure 1. The input data first goes through the convolution operation of the first convolution layer CONV1 to extract features and then goes through the ReLU activation function layer to convert the features into a set of feature maps and then goes through the pooling layer for maximum pooling, and downsampling the features, after the second repetition, connect the second pooling result with the fully connected layer, and finally output the result. Because the input data is one-dimensional, the size of the convolution kernel and the structure of the convolutional neural network (CNN) are simplified, and the network's computational cost is reduced. If you do not want to complicate your model's structure and make it tough to train, you should keep the kernel size constant in the convolutional layer. Original input data is derived from the TQE data. There are two convolutional layers: the first has 6 convolution kernels with a stride of 4, and the second has 12 convolution kernels with a stride of 10, and the convolution kernel size is 1. Each layer's pooling area is set to the same size, and the step size is 2, for the pooling layer, as shown in Figure 2. The process of selecting parameters is in the experimental part.

After determining the size and step size of the convolution kernel and the pooling area, the size of the output data after the convolution layer and the pooling layer can be obtained based on the calculation formula according to the input data. In the convolutional layer, assuming that the size of the input data volume is *W*_1_ × *H*_1_ × *D*_1_, the number of convolution kernels *K*, the size of the convolution kernel *S*, the step length *L*, and whether it has zero padding *P*, etc. parameters, the following formula calculates the output data *W*_2_ × *H*_2_ after the convolution layer; the specific formula is as follows:

(8) $$\begin{array}{c} W_{2}=\frac{W_{1}-S+2P}{L}+1, \end{array}$$

(9) $$\begin{array}{c} H_{2}=\frac{H_{1}-S+2P}{L}+1, \end{array}$$

(10) $$\begin{array}{c} D_{2}=K. \end{array}$$

In the same way, assuming that the size of the input data volume is *W*_1_ × *H*_1_ × *D*_1_ in the pooling layer, the maximum pooling downsampling operation of the pooling layer can be determined according to the size of the pooling area *S* and the step size *L*. The output data *W*_2_ × *H*_2_ × *D*_2_ were obtained later; the specific formula is as follows:

(11) $$\begin{array}{c} W_{2}=\frac{W_{1}-S}{L}, \end{array}$$

(12) $$\begin{array}{c} H_{2}=\frac{H_{1}-S}{L}, \end{array}$$

(13) $$\begin{array}{c} D_{2}=D_{1}. \end{array}$$

When the dimension of the input data is known to be one-dimensional and the size is known and according to the parameters set by each layer in the CNN structure, the final output data formed can be obtained by calculation.

#### 3.2.3. Model Training Process

The CNN model's training method is divided into two parts: forward propagation and back propagation. Forward propagation is used to build the CNN structure, while back propagation is used to finish the CNN model's training. The chain rule is mostly used in backpropagation, also known as error backpropagation, to compute the derivative value of the objective function in relation to the ownership value layer by layer from the back to the front, and compare the output result with the target value already given in the training set to obtain the error value. A threshold is specified in the neural network model. When the error value exceeds this threshold, the weights of each layer will be modified until the weights converge, and the training of the model ends. Therefore, this paper will solve the problem layer by layer from the back to the front from the CNN structure.

*(1) Reverse Derivation of the Fully Connected Layer*. In the fully connected layer, first calculate the derivative of the objective function *E* based on the last logits value of the network *t*^*l*+1^. The following formulas are shown:

(14) $$\begin{array}{c} \frac{\partial E}{\partial t^{l+1}}=\overset{m}{\underset{k=1}{\sum }}V_{k}R_{k}-V_{k}, \end{array}$$

(15) $$\begin{array}{c} t^{l+1}=wx^{l}+p, \end{array}$$

where *V* represents the one-hot vector, *l* represents the feature vector layer, *l* + 1 represents the output layer, *x*^*l*^ represents the output of the *l*th layer, *w* is the weight, and *p* is the bias.

During backpropagation, the error varies as the bias *p* of the neuron changes, so the error can be thought of as the sensitivity of *p*, the derivative of the error with respect to the basis. The derivative of the objective function *E* with respect to the fully connected layer weight *w* and the bias *p* can be expressed as

(16) $$\begin{array}{c} \frac{\partial E}{\partial w^{l}}=\frac{\partial E}{\partial t^{l+1}}∙\frac{\partial t^{l+1}}{\partial w^{l}}=\frac{\partial E}{\partial t^{l+1}}∙e^{l}, \end{array}$$

(17) $$\begin{array}{c} \frac{\partial E}{\partial p^{l}}=\frac{\partial E}{\partial t^{l+1}}∙\frac{\partial t^{l+1}}{\partial w^{l}}=\frac{\partial E}{\partial t^{l+1}}∙e^{l}. \end{array}$$

The activation function used in this paper is the ReLU function, so the derivative of the objective function *E* and ReLU is calculated as

(18) $$\begin{array}{c} \frac{\partial E}{{\partial e}^{l}}=\sum \frac{\partial E}{\partial t^{l+1}}∙\frac{\partial t^{l+1}}{{\partial e}^{l}}=\sum \frac{\partial E}{\partial t^{l+1}}∙w^{l}, \end{array}$$

(19) $$\begin{array}{c} \frac{\partial E}{\partial t^{l}}=\frac{\partial E}{{\partial e}^{l}}∙\frac{{\partial e}^{l}}{\partial t^{l}}=\left\{\begin{array}{c} 0,\;e^{l}\leq 0,\\ \frac{\partial E}{{\partial e}^{l}},\;e^{l}>0. \end{array}\right. \end{array}$$

The final objective function *E* is based on the derivative of the weight *w* in the fully connected hidden layer and the bias *p*, which can be obtained by substituting the result obtained from formula (19) into formulas (16) and (17).

*(2) Reverse Derivation of the Pooling Layer*. Since it is back propagation, after the derivative of the weight and bias of the objective function *E* is obtained in the fully connected layer, the derivative of the objective function with respect to each parameter in the pooling layer is then calculated. Unlike the fully connected layer, there are no weights in the pooling layer, so only the derivative of the neuron is calculated. The pooling layer uses maximum pooling, and only the maximum value in the region is retained during forward propagation. Therefore, during back propagation, the derivative is only passed to the neuron with the maximum value *N*_max_, and the rest of the neurons are discarded due to the fact that the derivatives are all 0, and the specific formula is

(20) $$\begin{array}{c} \frac{\partial E}{{\partial e}^{l}}=\frac{\partial E}{\partial V^{l}}∙\frac{\partial V^{l}}{{\partial e}^{l}}=\left\{\begin{array}{c} 0,\;N\neq N_{\max},\\ \frac{\partial E}{\partial V^{l}},\;N=N_{\max}. \end{array}\right. \end{array}$$

*(3) Reverse Derivation of the Convolutional Layer*. For the convolutional layer, the error is passed from the pooling layer, which is actually the reverse process of the downsampling operation. First, the derivative of the objective function with respect to each logits value is calculated. The specific formula as follows:

(21) $$\begin{array}{c} \frac{\partial E}{\partial y^{l}}=\frac{\partial E}{{\partial e}^{l}}∙\frac{{\partial e}^{l}}{\partial y^{l}}=\left\{\begin{array}{c} 0,\;y^{l}\leq 0,\\ \frac{\partial E}{{\partial e}^{l}},\;y^{l}>0. \end{array}\right. \end{array}$$

*(4) Parameter Update*. During back-propagation, after the parameters in the fully connected layer, activation function layer, pooling layer, and convolutional layer are, respectively, derived, each parameter needs to be updated, and finally, the update of the network model is completed. For the fully connected layer, the update formula of its weight *w* and bias *p* can be expressed as

(22) $$\begin{array}{c} w=w-\lambda \frac{\partial E}{\partial w}, \end{array}$$

(23) $$\begin{array}{c} p=p-\lambda \frac{\partial E}{\partial p}. \end{array}$$

After the parameters are updated, the samples will be input into the updated CNN model again, and the cycle will repeat until the model reaches the iterative condition or when it converges, and the training is terminated to complete the training of the CNN model. The final model is the trained CNN model.

### 3.3. Constructing a Quality Assessment System for Music and Art Teaching

There are two main methods of classroom TQE that are often used in colleges and universities. One is for the purpose of reward and punishment. In this kind of evaluation, the purpose is to promote teaching reform. The results of the evaluation directly determine the dismissal, demotion, promotion, dismissal, salary, bonus, and other personnel decisions of teachers; the disadvantage of this kind of evaluation is that it is a top-down evaluation that will only cause reactions and attention to a few people. The second goal is to help instructors improve their skills via assessment and professional development. Teachers' professional growth is the focus of this kind of review, which is also known as a developmental evaluation. There are no restrictions attached to rewards or penalties. The primary objective is to help college and university music instructors improve their skills and accomplish their ultimate goal of educating students in music. Under the developmental evaluation system, teachers can eliminate their concerns, because the results have little to do with rewards and punishments, they can evaluate more frankly, and teachers can accept the evaluation results more calmly. Teachers' morality and style, students' assessment and reflection of teachers' teaching, school teaching reform and teaching management information management, and strategies to enhance teachers' teaching quality are all included in the development evaluation of classroom teaching. The ultimate objective is to develop a scientific and fair framework for measuring teaching quality. In western countries, such as the US and the UK, more and more attention is paid to the use of development-oriented evaluation systems and methods. This is because developmental evaluation can improve the motivation of teachers' professional development, and evaluation can eliminate external rewards and punishments. Under such a mechanism, the progress of teachers' work will bring teachers a certain sense of achievement, self-awareness, and self-evaluation, so that teachers will put the improvement of the TQE in the first place, rather than simply pursuing external rewards and punishments. This research combs the domestic and foreign related researches on TQE and music art classroom TQE in colleges and universities by consulting relevant books, academic journals, network materials, etc. Based on the analysis of the current situation of TQE in the activity, a set of suitable teaching index evaluation system was designed, as shown in Table 1.

## 4. Experiment and Analysis

### 4.1. Data Source and Parameter Selection

In order to meet the TQE model designed, this paper designs a teaching evaluation data set according to the evaluation index system in Chapter 3, which contains 1000 sets of data, of which 800 sets are used as training sets and 200 sets are used as test sets. At present, the parameter determination of CNN still lacks a clear guiding theory and still relies on manual experience. The parameters must be constantly adjusted and compared in order to get the best value for each one. There are two convolutional layers, two pooling layers, and one fully connected layer in this chapter's model, as shown in the figure. At present, the parameter adjustment of neural network still relies on experience and constant comparison and adjustment for setting. The following is the comparison and selection process of some main parameters of the model.

## 5. Selection of Convolution Kernel and Step Size

In order to obtain the optimal number of convolution kernels and step size, this paper selects 8 combinations of convolution kernel and step size for experiments. The final result is shown in Figure 3. The results show that this paper chooses 20-4-10-1 parameter combination which is more advantageous.

## 6. Minibatch Parameter

The application of minibatch technology can improve the convergence speed of the model. The batch-size option specifies the number of samples utilized in a single training. When the batch size is too high, it is essentially the same as not employing minibatch technology; if a value is too little, the model will struggle to converge, resulting in poor fitting accuracy. This section selects 8 cases of 20, 40, 60, 80, 100, 120, 140, and 160, and sets a fixed number of 120 epochs to compare the convergence process. The experimental results are shown in Figure 4.

## 7. Model Parameter Verification Results

This paper uses Matlab to train the neural network, and the data training set and test set are divided according to 4 : 1. During the training process, each parameter selection is shown in Table 2. The number of training rounds is 50. During the training process, the accuracy of the training set and test set is shown in Figure 5:

### 7.1. Comparative Analysis of Results

This example takes the quality assessment of music and art teaching as an example and uses CNN model and back propagation (BP) neural network for prediction. The 15 evaluation indicators listed in Chapter 3 are the expected input. At the same time, the input data are normalised in order to make CNN training easier. The predicted values of 10 groups were selected to calculate the mean and plotted to observe. The results are shown in Figure 6.

The results show that the prediction accuracy of CNN is higher than that of BP network, and it is very close to the actual value. It can be shown that the network model proposed in this paper for the music and art TQE has very good performance.

## 8. Conclusion

The research on the TQE system of music art classroom teaching still needs to carry out research methods that are in-depth and systematic, combining theory and practice, so as to realize the key elements of music TQE in colleges and universities in essence. The current condition of music classroom teaching in colleges and universities is examined in this study, which includes an in-depth investigation of the elements affecting music education through inquiry and research on the current status of music classroom teaching. Construct the TQE system of music art based on the theoretical basis of TQE, and utilize the CNN network model to evaluate and produce satisfactory experimental results. The main work completed in this paper is as follows: (1) The basic situation of domestic and foreign research on music and art TQE is introduced, several commonly used TQE methods at home and abroad are analyzed, and the CNN neural network evaluation method is comprehensively introduced. (2) The CNN idea and network structure are explained, and a TQE system based on music art is built. (3) Using the trained CNN TQE model to conduct experiments and comparing it with back propagation neural network (BPNN), the final experimental results show that the method proposed in this paper has higher accuracy and better performance.

## Figures and Tables

**Figure 1:** Network structure diagram.

**Figure 2:** Network structure parameter diagram.

**Figure 3:** Convolution kernel number and step length experiment.

**Figure 4:** Minibatch parameters and their comparison.

**Figure 5:** Accuracy on training and test sets.

**Figure 6:** Comparison of predicted results of different models with actual results.

**Table 1:** Music and art teaching quality evaluation system.

First-level indicator	Secondary indicators	Label
Teaching preparation	Scientific and reasonable teaching design	X1
	Reasonable progress	X2
	Teaching plan writing specification	X3
Basic literacy	Rigorous teaching attitude and clear thinking	X4
	Vivid and accurate language	X5
	Good manners and appearance	X6
Teaching content	Combining theory with practice	X7
	Rich in content and appropriate information	X8
	Reflect the frontiers of the discipline	X9
Teaching method	Flexible method, suitable for course characteristics	X10
	Teaching students according to their aptitude	X11
	Use advanced teaching methods	X12
Teaching effect	Student attendance rate	X13
	Active classroom atmosphere	X14
	Complete teaching tasks with quality and quantity	X15

**Table 2:** Parameter selection during training.

Network depth	Mini-batch	Learning rate	Epochs	Training set	Test set
3	100	0.005	50	80%	20%

## Data Availability

The datasets used during the current study are available from the corresponding author on reasonable request.
